This article has been retracted.

# Regulation of the Proteasome by AMPK in Endothelial Cells: The Role of O-GlcNAc Transferase (OGT)

**DOI:** 10.1371/journal.pone.0036717

**Published:** 2012-05-04

**Authors:** Jian Xu, Shuangxi Wang, Benoit Viollet, Ming-Hui Zou

**Affiliations:** 1 Division of Endocrinology, Department of Medicine, University of Oklahoma Health Sciences Center, Oklahoma City, Oklahoma, United States of America; 2 Molecular Medicine, Department of Medicine, University of Oklahoma Health Sciences Center, Oklahoma City, Oklahoma, United States of America; 3 Inserm, U1016, Institut Cochin, Paris, France; 4 Cnrs, UMR 8104 Paris, France; 5 Université Paris Descartes, Paris, France; University of Hong Kong, China

## Abstract

26S proteasome is a macromolecular multi-subunit complex responsible for recognizing, unfolding, and ultimately destroying proteins. It remains poorly understood how 26S proteasome activity is regulated. The present study was to investigate if AMP-activated protein kinase (AMPK) functions as a physiological suppressor of the 26S proteasome in endothelial cells. 26S proteasome assembly, activity, and O-GlcNAcylation of P700 were assayed in cultured human umbilical vein endothelial cells (HUVEC) and mouse aortas isolated from C57BL6 wild type and AMPKα2 knockout mice with or without being exposed to selective AMPK activators or inhibitors. Pharmacological and genetic activation of AMPK effectively suppresses 26S proteasomes in endothelial cells. Conversely, inactivation of AMPK either pharmacologically or genetically increases 26S proteasome activity; furthermore, the inactivation decreases the O-GlcNAcylation of PA700/S10B (the regulatory complex in 26S proteasomes) and increases the assembly of 26S proteasomes. In contrast, AMPK activation increases levels of O-GlcNAcylated PA700/S10B, likely through enhanced association of PA700 with O-GlcNAc transferase (OGT), the enzyme that catalyzes protein O-GlcNAcylation. Finally, aortas from AMPK-KO vs wild type mice exhibit elevated 26S proteasome activity in parallel with decreased PA700/S10B O-GlcNAcylation and PA700/S10B-OGT association. Taken together, we conclude that AMPK functions as a physiological suppressor of 26S proteasomes.

## Introduction

The ubiquitin proteasome system (UPS) is the major non-lysosomal degradative machinery for most intracellular proteins [1], [2]. A key component of this machinery is the 26S proteasome [3], a macromolecular multi-subunit complex that is responsible for recognizing, unfolding, and ultimately destroying proteins. To be degraded, most target proteins must first be tagged with polyubiquitin chains, generally at the -NH_2_ group of an internal lysine residue [4], [5]. The 26S proteasome (a 2-MDa complex) is made up of two sub-complexes: the catalytic particle (or 20S proteasome) and the regulatory particle (19S proteasome) [3]. The 20S proteasome is a cylindrical protease complex consisting of 28 subunits configured into four stacks of heptameric rings. On the other hand, the 19S (or PA700) consists of at least 18 subunits, including 6 putative ATPases and 12 non-ATPase subunits [3], [6]. The 26S proteasome is known to require ATP hydrolysis to degrade ubiquitinated substrates and for its assembly [7]. Over the past few years, it has become clear that deregulation of the UPS leads to inappropriate destruction or accumulation of specific proteins and ensuing pathological consequences [1]. The UPS is now recognized as a regulator of the cell cycle and cell division [8], [9], immune responses and antigen presentation [10], [11], apoptosis [12], and cell signaling [13], [14]. The UPS has been shown to be either activated in certain cancers (e.g., multiple myeloma) [15], [16] or dysfunctional in neurodegenerative disorders (e.g., Alzheimer's disease, Huntington's disease [17], and amyotrophic lateral sclerosis [18], [19]).

AMPK was initially identified as a sensor of cellular energy [20], [21] and is also likely a sensor of cellular redox status [22], [23]. As a phylogenetically conserved enzyme, AMPK is present in all mammalian cells. AMPK is a heterotrimeric enzyme comprised of a catalytic (α) subunit and two regulatory (β and γ) subunits [24], [25]. AMPK is activated by at least three distinct signals: a Ca^2+^-dependent pathway mediated by calcium calmodulin-dependent kinase kinase-β (CaMKK-β) [26], an AMP-dependent pathway mediated by LKB1 [27], and TGF-β-activated kinase-1 (Tak1) [28] via phosphorylation at Thr172 on the α-subunit. Binding of AMP to the γ-subunit leads to allosteric activation of AMPK, a change that also protects the Thr172 site from dephosphorylation [29]. Once activated, AMPK switches on catabolic pathways that generate ATP, while switching off ATP-consuming processes (e.g., biosynthesis, cell growth, and proliferation). In this way, it functions as “energy gauge” [29], [30]. This has been regarded as a fundamental feature of multiple AMPK-mediated biological processes. AMPK is generally quiescent under normal conditions but is activated in response to hormonal signals and stresses sufficient to increase the AMP/ATP ratio, such as hypoglycemia, strenuous exercise, anoxia, and ischemia.

In contrast to traditional *N*- and *O-*glycosylation, which occurs in secretory pathways (endoplasmic reticulum and Golgi) [31], O-GlcNAcylation is defined as the *O*-linked attachment of *N*-acetylglucosamine (*O-Glc*NAc) onto Ser/Thr residues of cytosolic and nuclear proteins [32]. O-GlcNAcylation is an important regulatory mechanism for signal transduction [32], [33], [34], [35]. OGT mediates O-GlcNAcylation, while removal of O-GlcNAc is catalyzed by the complementary β-N-acetylhexosaminidase (O-GlcNAcase, or OGlcNAc hydrolase as OGA). To date, more than 80 different proteins including transcription factors, kinases, phosphatases, cytoskeletal proteins, nuclear hormone receptors, nuclear pore proteins, signal transduction molecules, and actin regulatory proteins [34], [35] have been shown to undergo O-GlcNAcylation [35] although the mechanisms underlying OGT regulation are not completely understood.

Endothelial dysfunction, which is characterized by impaired endothelium-dependent vasorelaxation [36], [37], [38], is a common feature of CVD. During CVD, the endothelium losses its homoeostatic potential to inhibit the disease process [38]. We [39], [40], [41] and others [42] have shown that the UPS can contribute to the development of endothelial dysfunction, which is reflected as enhanced 26S proteasome activity, an accelerated degradation of endothelial-protective molecules (such as the guanosine 5-triphosphate cyclohydrolase I or GTPCH I, the rate limiting enzyme essential for the de novo synthesis of an eNOS co-factor [39], [40], [43]), and consequent impaired endothelium-dependent vasorelaxation. Most importantly, we have discovered that such an impairment can be restored by activation of AMPK [43]. Interestingly, we recently found that global knockout of both AMPK and ApoE genes enhances NAD(P)H oxidase expression as well as exacerbates atherosclerosis and endothelial dysfunction by influencing 26S proteasome activation [44]. Further, we found that AMPK activation alleviates diabetic endothelial dysfunction by suppressing the 26S proteasome [43]. However, how AMPK regulates 26S proteasome activity in these cases remains unknown. Here we report that AMPK suppresses 26S proteasome activity by promoting PA700/S10B-OGT association and PA700/S10B O-GlcNAcylation.

## Materials and Methods

### Materials and animal model

Mouse-derived PA700/S10B antibody was from Abcam (Cambridge, MA); MG132 from BioMol (Plymouth Meeting, PA); fluorogenic proteasome substrates from Calbiochem (San Diego, CA); Proteasome inhibitor MG132 was purchased from BioMol (Plymouth Meeting, PA). 1% protease inhibitor cocktail were obtained from Sigma (St Louis, MO). 1% phosphatase inhibitor cocktail was purchased from Pierce. PUGNAc (O-GlcNAcase inhibitor) was from Sigma (St Louis, MO). Anti-O-GlcNAc antibody (CTD110.6 antibody, sc-59623) and negative control siRNA or target-specific siRNA duplex against OGT were from Santa Cruz Biotechnology (Santa Cruz, CA). Control siRNA duplex and PA700-specific siRNA duplex were from Ambion (Austin, TX). Protein-A Sepharose CL-4B was purchased from Amersham Biosciences (Piscataway, NJ). All other chemicals were obtained from Fisher Scientific (Pittsburgh, PA), unless otherwise noted, were of the highest possible grade. Human umbilical vein endothelial cells (HUVEC) were obtained from Cascade Biologics (Walkersville, MD).

Control and AMPKα2^−/−^ male mice were studied at 12 weeks of age. The establishment and characterization of AMPKα2^−/−^ mice were previously reported [45]. Animals were housed under controlled temperature (21°C) and lighting, with 12 hours of light and 12 hours of dark, and had free access to water and a standard mouse chow diet. All procedures were approved by the University of Oklahoma Health Sciences Center Institutional Animal Care and Use Committee (IACUC Protocol: 10-005).

### 26S proteasome activity assay

26S proteasome function was assayed as described previously but with minor modifications [46]. Chymotrypsin-like activity was measured using SucLLVY-7-amido-4-methylcoumarin (AMC), trypsin-like activity with Bz-VGR-AMC, and caspase-like activity with Z-LLE-AMC. These fluorogenic proteasome substrates were added to the cell lysate at a final concentration of 80 µM in 1% DMSO. ATP-dependent cleavage activity was monitored continuously by detection of free 7-amido-4-methylcoumarin using a fluorescence plate reader (Gemini, Molecular Devices) at 380/460 nm at 37°C.

### Adenoviral infection and siRNA transfection

Confluent HUVEC were infected with adenovirus encoding AMPK-CA, AMPK-DN, or GFP (as adenoviral infection control), as described previously [43]. SiRNA transfection was done, as described previously [40].

### Identification of O-GlcNAc-modified proteins in mouse aortas

Aortas isolated from mice were weighed and homogenized in lysis buffer containing 25 mmol/L HEPES (pH 7.0), 1 mmol/L EDTA, 1 mmol/L EGTA, 1% NP-40, 0.1% SDS, 1% protease inhibitor cocktail (Sigma, St Louis, MO), 1% phosphatase inhibitor cocktail, and 1–100 µmol/L PUGNAc (O-GlcNAcase inhibitor). Proteins modified by O-linked GlcNAc will be immunoprecipitated with anti-O-GlcNAc antibody. Proteins were released from the beads by boiling in Laemmli buffer containing 50 mmol/L dithiothreitol and separated by 12% SDS-PAGE. Separated proteins were subjected to western blot analysis using anti-PA700 antibodies.

### Statistical analysis

Statistical comparisons of all results were analyzed using a one-way ANOVA. Values are expressed as mean ± SEM. p<0.05 is considered as significant.

## Results

### AMPK inactivation increases 26S proteasome activity in HUVEC

To determine whether AMPK inactivation alters proteasome activity, we tested the effect of modulating AMPK activity on proteasome activities in HUVEC. Compound C (0.5 µmol/L for 15 min), the nonselective inhibitor of AMPK [47], but not vehicle (DMSO), significantly increased 26S proteasome activity, and this effect could be reversed by co-incubation with MG132 (proteasome inhibitor, 0.5 µmol/L) or AICAR (5-aminoimidazole-4-carboxamide ribose, an AMPK activator) (Fig. 1A). As expected, MG132 alone significantly inhibited proteasome activity (Fig. 1A). However, AICAR alone for 6 h had no significant effect on 26S proteasome activity (Fig. 1A), although prolonged incubation with AICAR (overnight) did suppress 26S proteasome activity in HUVEC [43].

**Figure 1:** AMPK suppression increases 26S activity in HUVEC. AMPK suppression in HUVEC either by (A) compound C (10 µmol/L for 2 hour) or by (B) overexpression of AMPK-dominant negative mutant (DN) increases 26S proteasome activities, as demonstrated by ATP-dependent increased chymotrypsin-like, trypsin-like and caspase-like activity on fluorescent proteasome substrates. MG132 (0.5 µmol/L for 1 hour) or AICAR (2 mmol/L for 6 hours) treatment blocks the increased chymotrypsin-like activity in AMPK-suppressed HUVEC. * indicates P<0.05 vs vehicle (DMSO) or GFP, n = 3 per group.

Next, we investigated whether genetic inhibition of AMPK had a similar effect as pharmacological AMPK inhibition by compound C. Overexpression of an AMPK dominant negative mutant (AMPK-DN), but not of GFP (control), also induced 26S proteasome activation, while MG132 could block the activation (Fig. 1B). Interestingly, unlike MG132, AICAR failed to inhibit AMPK-DN promoted 26S proteasome activation (Fig. 1B), suggesting that the suppressive effect of AICAR on proteasome was mediated, at least in part, by AMPK activation. Together, these results suggest that AMPK inactivation contributes to 26S proteasome activation in HUVEC.

Of note, AMPK inactivation increased all 3 major protease-like activities at various degrees (Fig. 1A and B). However, only chymotrypsin-like activity could be significantly reversed or suppressed by the treatment with AICAR (Fig. 1A) or MG132 (Fig. 1A and B) at indicated concentrations and duration of the treatment. Therefore, we only used chymotrypsin-like activity to demonstrate AMPK dependent effects on 26S proteasome activity in subsequent cell experiments.

### AMPK inhibition-induced 26S proteasome activation is accompanied by increased 26S assembly

To confirm that AMPK responds to its activator or inhibitor as reported, we first detected AMPK activation in challenged HUVEC. As expected, AICAR promoted, but compound C suppressed AMPK phosphorylation (Thr172), a marker of AMPK activation, so as its downstream target ACC phosphorylation (Ser79), based on quantified data that had been normalized with the total AMPK or ACC protein levels (Fig. 2A). To begin to understand how AMPK inactivation may activate the 26S proteasome, we first determined if pharmacological or genetic inactivation of AMPK affects 26S assembly (association), an event known to be crucial for 26S proteasome activation [48], [49], [50]. Western blot analysis of PA700 immunoprecipitates using 20S proteasome-specific antibody (against its β7 subunit) revealed that a greater association occurred between PA700 and the 20S proteasome in compound C-treated cells than in vehicle-treated cells (Fig. 2B). However, co-incubation of cells with AICAR abolished the effect of compound C. None of these treatments altered either PA700 or β7 protein levels (Fig. 2B). To confirm the 26S proteasome assembly, we further separated the same samples under non-reducing condition on a native gradient PAGE (3–14%) and performed Western blot staining with antibodies to the subunits of either 19S (PA700/S10B) or 20S proteasome sub-complex (β7) on duplicate blots. As shown in Fig. 2C, on the same molecular weight site (above the native protein marker 1236 kD) of the duplicated blots, both staining for PA700/S10B and β7 were increased in the presence of compound C (Fig. 2C left), pre-incubation with AICAR blocked the increase (Fig. 2C), suggesting 26S proteasome assembly enhancement did occur in the cells. The enhanced 26S assembly was accompanied by an increase in 26S proteasome activity (Fig. 2D).

**Figure 2:** Increased 26S proteasome activity in AMPK-suppressed HUVEC is correlated with the enhanced association of 19S and 20S sub-complexes. Compound C (10 µmol/L for 2 hour)-treated HUVEC present (A) AMPK inactivation, (B) an increase in association of PA700/S10B (from 19S complex) with β7 (from 20S complex), which can be blocked by AICAR pre-incubation (2 mmol/L for 6 hours), (C) 26S proteasome assembly (same samples were run on 3–14% native-PAGE under non-reducing condition followed by conventional Western blot on duplicated blots with PA700/S10B and β7 antibodies, respectively), and (D) an increase in 26S proteasome activity (chymotrypsin-like) (n = 3). The increased association of proteasome sub-complex is also observed in (E) HUVEC overexpressing AMPK-DN but not AMPK-CA or GFP. All of the blots shown are representative of 3 independent experiments. NS represents not significant.

Finally, given the potential non-selective effects of compound C [47], we tested if AMPK-DN could replicate the effect of compound C. HUVEC overexpressing AMPK-DN showed enhanced 26S assembly compared to those overexpressing GFP (control) or constitutively active AMPK (AMPK-CA) (Fig. 2E). Of note, none of these treatments affected PA700 or the β7 protein levels (Fig. 2E). Like in compound C-treated cells, the increased 26S proteasome assembly (association) in AMPK-DN overexpressing HUVEC was accompanied with an increase in 26S proteasome activity (Fig. 1B), in contrasting to the suppressive effect on 26S proteasome activity detected in AMPK-CA over-expressing HUVEC [43]. The fact that 26S activation could always be detected no matter how AMPK was inactivated suggests that AMPK regulates 26S proteasomes.

### AMPK activation increases OGT-PA700 association and PA700 O-GlcNAcylation, while AMPK inactivation decreases these outcomes

Next, we investigated whether modulation of AMPK activity could alter the OGT-PA700 association and PA700 O-GlcNAcylation. Western blot analysis of OGT immunoprecipitates using specific PA700 antibody showed that compound C reduced OGT-PA700 association, and this effect was reversed by AICAR (Fig. 3A), consistent with the ability of compound C to decrease PA700 O-GlcNAcylation in an AICAR-reversible manner (Fig. 3A).

**Figure 3:** AMPK suppression is accompanied by the decreased association of OGT with proteasome. AMPK suppression in HUVEC either by (A) compound C (10 µmol/L for 2 hour) or by (B) overexpression of AMPK-dominant negative mutant (DN) decreases both the OGT association with proteasome and the O-GlcNAcylation of PA700/S10B (vs. controls), which can be reversed by AICAR pre-incubation (2 mmol/L for 6 hours) in AMPK-present but not AMPK-DN cell. In contrast, constitutive activation of AMPK (overexpression of AMPK-CA vs GFP) (B) increases OGT-PA700 association. All of the blots shown are representative of 3 independent experiments. NS reprents not significant.

We also tested if genetic inhibition of AMPK through overexpression of AMPK-DN produced a similar effect as compound C. Compared to GFP overexpression, AMPK-DN overexpression elicited a dramatic reduction in OGT-PA700 association (Fig. 3B), which might contribute to enhanced 26S proteasome assembly (Fig. 2C) and activation (Fig. 2D). Importantly, although AICAR increased the association of inhibitory OGT with PA700 in cells overexpressing GFP (Fig. 3B), this effect was absent in cells overexpressing AMPK-DN (Fig. 3B), indicating that AMPK participated in enhanced OGT-P700 association. Conversely, constitutive activation of AMPK (overexpression of AMPK-CA) resulted in greater OGT-PA700 association than GFP overexpression (Fig. 3B). However, none of the treatments altered the protein levels of PA700 or OGT (Fig. 3B).

### An OGT activator, but not an OGA inhibitor, blocks 26S proteasome activation induced by AMPK inhibition

To determine if OGT mediates AMPK suppression of proteasome activity, we compared 26S proteasome assembly in the presence of UDP-GlcNAc, a specific OGT substrate and activator. Western blot analysis of PA700/S10B immunoprecipitates by using specific 20S proteasome antibody (to its β7 subunit) revealed that activation of OGT by UDP-GlcNAc blocked compound C-induced increases in 26S proteasome assembly (Fig. 4A) and activation (Fig. 4B). OGT treatment also inhibited the decrease of PA700/S10B O-GlcNAc modification (Fig. 4A). Two dynamic enzymes directly control O-GlcNAcylation: OGT, which catalyzes O-GlcNAcylation, and its negative regulator OGA, which removes O-GlcNAc. Inhibition of OGA has been shown to have synergistic effects on OGT activation [34]. We investigated whether OGA, like OGT, participates in AMPK regulation of the 26S proteasome. Surprisingly, inhibition of OGA with PUGNAc did not prevent compound C-enhanced 26S proteasome assembly, reduction of PA700/S10B O-GlcNAcylation (Fig. 4A) or activation (Fig. 4B). To confirm the functional outcomes of altered 26S proteasome activity, we measured the protein levels GTPCH I, which degradation is enhanced by 26S proteasome activation [39], [40], [43]. As depicted in Fig. 4, 26S proteasome activation by compound C reduced GTPCH I protein levels (Fig. 4); pre-incubation of OGT activator UDP-GlcNAc, but not OGA inhibitor PUGNAC, blocked the reduction of GTPCH I (Fig. 4C). Collectively, these data indicate that OGT plays a major role in AMPK regulation of the proteasome.

**Figure 4:** Activation of OGT prevents AMPK-inhibition induced 26S proteasome activation. AMPK suppression by compound C (10 µmol/L for 2 hour) in HUVEC (A) increases the association of PA700/S10B (from 19S complex) with β7 (from 20S complex) accompanied by a decrease of PA700/S10B O-GlcNAc modification, and (B) increases 26S proteasome activity, which can be prevented by pre-incubation of UDP-GlcNAc (25 µmol/L for 30 min), but not by PUGNAc (14 µmol/L for 30 min), the inhibitor of O-GlcNAcase. The blots shown are representative of 3 independent experiments.

### siRNA-mediated knockdown of OGT enhances 26S proteasome assembly and activity

To determine whether OGT is required for 26S proteasome regulation by AMPK, we performed knockdown experiments using siRNA. We repeated the experiments previously shown in cells infected with siRNA. As shown in Fig. 5, OGT protein levels were more than 90% lower in cells transfected with OGT siRNA than in control siRNA-treated cells. Surprisingly, knockdown of OGT significantly increased 26S assembly, as reflected by an increase in PA700 and β7 association (Fig. 5A), and 26S proteasome activity (Fig. 5B). However, compound C did not further enhance 26S proteasome assembly (Fig. 5A) and activity (Fig. 5B) in OGT siRNA-transfected cells as it did in control siRNA cells (Fig. 5A and B). The absence of this effect in OGT knockdown cells further suggests that OGT is indispensable for AMPK regulation of the 26S proteasome. As shown for other treatments, these treatments did not alter PA700 or β7 protein levels (Fig. 5A). Cumulatively, these results suggest that, under basal conditions, AMPK serves to keep the 26S proteasome at the minimal required activation level by maintaining the association of OGT with PA700 and in turn, keeping O-GlcNAcylation of PA700 in a constitutive state.

**Figure 5:** Loss of OGT increases 26S proteasome assembly. HUVEC transfected with OGT siRNA but not control siRNA show an increase in (A) association of PA700/S10B (from 19S complex) with β7 (from 20S complex) and (B) 26S proteasome activity, mimicking the effect of AMPK-suppression by compound C (10 µmol/L for 2 hour). The blots shown are representative of 3 independent experiments. * represents p<0.05 vs the control (without compound C treatment).

### Aorta from AMPK-KO mice exhibit a decrease in OGT-PA700/S10B association along with an increase in 20S complex formation and 26S proteasome activity

We next explored if AMPK regulates the 26S proteasome *in vivo*. We compared aortic proteins prepared from AMPKα2-KO and WT (C57BL/6J) mice. Western blot analysis revealed that, although AMPKα2 protein was undetectable in AMPKα2-KO aortas (Fig. 6A), levels of β-actin (Fig. 6A), OGT (Fig. 6B), β7 (Fig. 6C) and PA700/S10B (Fig. 6) did not significantly differ between WT and AMPK-KO aortas. However, compared to WT aortas, AMPK-KO aortas exhibited a decrease in OGT-PA700/S10B association (Fig. 6B), an increase in 26S assembly as seen by an increase in PA700/S10B-β7 association (Fig. 6C), and an increase in all three major protease-like activities of the 26S proteasome (Fig. 6D).

**Figure 6:** AMPK depletion is associated with decreased association of OGT with proteasome and increased 26S proteasome assembly and activity in AMPK-KO mice. Gender (male) and age (12 weeks) matched mice (n = 8/group) with the genotypes of wild type (C57BL/6J) and AMPKα knockout were used. Compared to aortas from wild type (C57BL/6J) mice, (A) aortas from AMPKα knockout mice exhibit (B) a decrease in the association of OGT with proteasome (PA700/S10B), (C) an increase in proteasome assembly (PA700/S10B-β7 association), and (D) an increase in 26S proteasome activity, without alteration in the expression levels of proteasome (β7 or PA700/S10B) or OGT. * represents p<0.05 vs wild type (n = 8).

## Discussion

The present study has demonstrated that inactivation of AMPK elevates 26S proteasome activity and that this effect is associated with decreased PA700/S10B O-GlcNAcylation and increased 26S proteasome assembly. Conversely, AMPK activation increases GlcNAcylated PA700/S10B by stabilizing its association with OGT, the key enzyme responsible for protein O-GlcNAcylation. OGT appears to be crucial for this event, as AMPK-mediated 26S proteasome inhibition is blocked by siRNA-mediated OGT knockdown. The most conclusive evidence that AMPK suppresses the 26S proteasome comes from analysis of aortas from AMPK-knockout (AMPK-KO) mice. We found that, compared to wild type (WT) aortas, aortas from AMPK-KO mice exhibit elevated 26S proteasome activity with decreased PA700/S10B O-GlcNAcylation and PA700/S10B-OGT association. Importantly, in spite of different mechanisms underlying AMPK inactivation by compound C and AMPK-DN, both treatments in HUVEC induce 26S proteasome activation, indicating the essential role of AMPK activity in 26S proteasome regulation. Furthermore, all the promoted 26S proteasome activations through AMPK suppression in HUVEC are attenuated by MG132, a potent proteasome inhibitor, suggesting AMPK suppression is truly associated with 26S proteasome activation. Overall, our results support the notion that AMPK, a sensor of cellular energy, maintains low basal 26S proteasome activity by keeping PA700/S10B O-GlcNAcylated and in turn, suppressing 26S proteasome activity and likely preventing 26S proteasome-mediated degradation of endothelial protective molecule(s).

In contrast to traditional *N*- and *O-*glycosylation, which occurs in secretory pathways (endoplasmic reticulum and Golgi) [31], O-GlcNAcylation is defined as the *O*-linked attachment of *N*-acetylglucosamine (*O-Glc*NAc) onto Ser/Thr residues of cytosolic and nuclear proteins [32]. O-GlcNAcylation is an important regulatory mechanism for signal transduction [32], [33], [34], [35]. OGT mediates O-GlcNAcylation, while removal of O-GlcNAc is catalyzed by the complementary β-N-acetylhexosaminidase (O-GlcNAcase, or OGlcNAc hydrolase as OGA). To date, more than 80 different proteins including transcription factors, kinases, phosphatases, cytoskeletal proteins, nuclear hormone receptors, nuclear pore proteins, signal transduction molecules, and actin regulatory proteins [34], [35] have been shown to undergo O-GlcNAcylation [35] although the mechanisms underlying OGT regulation are not completely understood.

The most important finding of this paper is that we demonstrate that OGT and its connection to the AMPK-mediated regulation of 26S proteasome in endothelial cell. The present study demonstrates that AMPK, as a physiological suppressor of 26S proteasome, regulates proteasome function by controlling OGT-mediated proteasome O-GlcNAcylation. Indeed, there is evidence that 19S subunit can be subjected to O-GlcNAcylation with consequent 26S proteasome inhibition [51]. Hence, O-GlcNAc is considered an endogenous inhibitor of the 26S proteasome [51]. A proteomic study revealed that several other proteins in the 26S proteasome can also be extensively O-GlcNAcylated [52]. Hence, O-GlcNAc is considered an endogenous inhibitor of the 26S proteasome [51] and O-GlcNAc modification links a nutritional sensor to modulation of proteasome function [53]. Intriguingly, AMPK, a cellular energy sensor and a major component of the nutrient pathway [54], has recently been linked to O-GlcNAc modification through OGT upregulation [55]. This effect is likely independent of a direct association between OGT and AMPK [56], though co-immunoprecipitation of these proteins is possible [57]. In line with this relationship, we found that OGT is essential in mediating AMPK-dependent 26S proteasome suppression both in cultured cells and aortas of AMPK2α-KO mice, likely through the control of PA700/S10B modification. These data suggest that a novel functional link exists between AMPK and OGT that regulates 26S proteasome function in endothelial cell.

It is worthy of note that compared to the effect of AMPK-DN, AMPK-CA alone did not generate a robust changes in 26S proteasomes assembly. This is in line with the observations that AMPK-CA alone has either marginal [43], [44] or not significant effects on 26S proteasome activity. All these data might imply that basal AMPK activity is essential in keeping 26S proteasome activity in check; further studies are warranted.

The concept that AMPK activation could be used as a strategy to promote vascular health, including overcoming endothelial dysfunction, has only recently emerged [22], [58], [59]. Endothelial dysfunction, characterized by impaired endothelium-dependent vasorelaxation, is a common feature of CVD including diabetes and hypertension. We have recently shown that link exists between 26S proteasome activation and endothelial dysfunction through accelerated proteasomal degradation of GTP-CH I and consequent BH4 deficiency [39], [40]. More importantly, we have demonstrated that activation of AMPK by Metformin reverses endothelial dysfunction in a 26S proteasome-dependent fashion in streptozotocin-induced diabetic mice [43]. Thus, our data suggest that AMPK-dependent OGT-mediated 26S proteasome suppression might operate *in vivo* contributing to the protective effect of AMPK on endothelial function in our previous studies [43], [44] In summary, this is the first report of a novel function for AMPK-dependent 26S proteasome regulation in endothelial cells, a mechanism that may bridge endothelial function with both the energy (AMPK) and metabolic (OGT) sensors.
